# Application Effect of the Standard Operating Procedure in the Prevention of Venous Thromboembolism

**DOI:** 10.1155/2022/5019898

**Published:** 2022-01-07

**Authors:** Hongxia Zhang, Zonghong Zhu, Xiaoyan Wang, Xiaofeng Wang, Limin Fan, Ranran Wu, Chenjing Sun

**Affiliations:** ^1^Department of Neurology, The Sixth Medical Center of PLA General Hospital, Beijing 100048, China; ^2^Department of Emergency, The Sixth Medical Center of PLA General Hospital, Beijing 100048, China; ^3^Department of Rehabilitation Medicine, The Southern Medical Branch of PLA General Hospital, Beijing 100071, China

## Abstract

**Objective:**

To investigate the application effect of the standard operating procedure (SOP) in the prevention of venous thromboembolism (VTE).

**Methods:**

The clinical data of patients admitted to respiratory, cardiovascular, neurological, and geriatric departments in the hospital (November 2020–May 2021) were retrospectively analyzed, and the patients in line with the inclusion criteria were equally randomized into the observation group (OG) and the control group (CG). The CG was treated with the routine nursing, and the OG received the SOP of VTE prevention additionally. After the record of the incidence of VTE and nursing satisfaction of the two groups, scores of VTE awareness were compared.

**Results:**

One hundred and twenty patients were included in this study, and no obvious difference was found in the general data of patients (*P* > 0.05). Compared with the CG, the incidence of VTE of the OG was obviously lower (*P* < 0.05). After nursing, compared with the CG, scores of VTE awareness in the OG were conspicuously higher (*P* < 0.001), and scores of VTE awareness of the nursing staff were conspicuously higher than those before nursing (*P* < 0.001). Compared with the CG, nursing satisfaction of the OG was obviously higher (*P* < 0.001).

**Conclusion:**

SOP can reduce the incidence of VTE of patients, improve their disease awareness, and enhance their nursing satisfaction, which should be popularized in practice.

## 1. Introduction

Venous thromboembolism (VTE) is known as the venous reflux disorder, referring to a condition in which a blood clot forms in the deep veins (known as deep vein thrombosis, DVT) and in the lungs (known as pulmonary embolism, PTE) [1, 2]. Epidemiological reports show that VTE has a very high mortality rate and disability rate, which is one of the most common complications of hospitalized patients in the internal medicine department [3]. Patients may have pulmonary thromboembolism and venous gangrene in the early stage and may present with repeated swelling, itching, and ulceration of lower limbs in the later stage. Some patients even face the risk of amputation [4, 5]. Meanwhile, VTE prolongs the hospitalization time, increases medical expenses, and leads to death or disability for patients [6], while many studies have confirmed that the incidence of VTE can be reduced by 60% through preventive nursing [7]. Therefore, it is urgent to further explore the early prevention and standardized treatment of VTE. At present, VTE prevention management system has been tried in some hospitals in China, but there is no unified standard, so it can only be carried out in the way of the thrombosis specialist group [8, 9]. The effectiveness, timeliness, and scientificity of the VTE prevention system are expected to be improved.

Reviewing the literature at home and abroad, standard operating procedure (SOP) is often used in first aid and intensive care [10]. This nursing method aims to refine and quantify the standard operating steps, so as to guide the daily work and improve the nursing systematicness, standardization, and operability [11]. SOP can provide nursing staff with a unified format for VTE prevention so that they can carry out prevention work under the specific and clear guidance, in place of the previous experience-based care [12]. There are no studies to apply the SOP in VTE prevention currently. Therefore, this paper introduces the SOP into VTE prevention for hospitalized patients in internal medicine by reviewing the literature and guidelines combined with clinical experience, summarized as follows.

## 2. Materials and Methods

### 2.1. Research Design

This retrospective study was conducted in the hospital (November 2020–May 2021) to explore the application effect of the SOP in the prevention of VTE. As a double-blind study, neither the study subjects nor the investigators were aware of the trial grouping, and the study designer was responsible for arranging and controlling the whole trial.

### 2.2. Research Subjects

The clinical data of patients admitted to respiratory, cardiovascular, neurological, and geriatric departments in the hospital (November 2020–May 2021) were retrospectively analyzed. The inclusion criteria were as follows: (1) the scores of Padua [13] of patients were ≥4 or D-dimer (D-D) level was increased. (2) Patients received the whole treatment in the hospital, and no one was transferred to other hospitals halfway. (3) No DVT was observed in patients after examination by using the color Doppler ultrasound instrument. (4) The hospitalization time of patients was ≥3 days. (5) Patients were at the age of 18 and above. The exclusion criteria were as follows: (1) patients could not be communicated with due to hearing impairment, language impairment, unconsciousness, or mental illness. (2) Patients withdrew halfway. (3) Patients had severe organic diseases.

### 2.3. Procedures

The procedures of the study are shown in Figure 1.

### 2.4. Moral Consideration

The study was in accordance with the principles of Declaration of Helsinki (2013) [14]. After enrollment, the research subjects were informed of the purpose, significance, content, and confidentiality of the study and signed the consent form.

## 3. Methods

The CG received routine nursing (basic prevention, drug prevention, and mechanical prevention). (1) Basic prevention: basic health education was given to patients to enhance their awareness on VTE prevention. Patients were encouraged to exercise regularly, such as ambulation in the morning and ankle exercises in bed. Patients were asked to drink more water, with the water intake of 1500–2000 ml daily. Patients who took dehydrating drugs and had more perspiration should be rehydrated promptly to maintain effective circulating blood volume. Venipuncture should be away the hemiplegic side and lower limbs. (2) Drug prevention: if necessary, patients should be treated with low-molecular-weight heparin, unfractionated heparin, and anticoagulant. (3) Mechanical prevention: it included graduated compression stockings, and pneumatic cyclic actuation device was used, and it could not be applied in patients with contraindications to mechanical prevention, local gangrene, acute dermatitis, severe deformity, and peripheral vascular diseases.

The OG was treated with the SOP of VTE prevention. (1) Evidence-based nursing was adopted. After fully understanding the SOP of VTE prevention, nursing scheme was formulated by using Chinese and English databases and online resources, extensively reading the literature, and combining with the actual situation of patients. (2) The risk assessment of VTE was performed in all patients after admission. ① Disease condition of patients was evaluated and recorded within 24 hours after admission. ② The risk of VTE was assessed by the Padua prediction score. ③ The responsible nurses were responsible for information acquisition. 0–3 points indicated low risk, 3 points indicated middle risk, and more than 3 points indicated high risk. ④ Basic precautions were given to low-risk patients, while high-risk patients as well as those who stayed in bed for ≥3 days were observed for the VTE symptoms, and leg circumference was measured along with performing bedside B-ultrasound examination (SonoScape Medical Co., Ltd.; Medical Products Administration of Guangdong Province, approval no. 20082230416) in the case of the presence of VTE outside the hospital. The responsible nurses were responsible for informing doctors of the results and took corresponding nursing precautions. ⑤ After risk assessment by doctors, mechanical prevention and drug prevention were used for patients with no or low risk of bleeding, and mechanical prevention was used for patients with high risk of bleeding. ⑥ Warning signs were made according to the risk levels, and the bedside card was marked with corresponding color, with high-risk warning cards for high-risk patients. (3) According to the risk levels, corresponding nursing precautions were carried out for patients. Health education was performed during the whole hospitalization including basic introduction of VTE, the hazards of VTE, clinical manifestations of VTE, and precautions that need to be taken in the way of slides to enhance patients' awareness of the disease. ① Basic precautions were applied to all patients, and other precautions were performed based on VTE risk assessment. The specific operation was the same as that in the CG. (4) Quality evaluation. ① The thrombosis prevention evaluation form was established to record the implementation of preventive nursing measures, lower limb blood circulation, and daily leg circumference measurement. Patients with signs of DVT were given timely treatment in the case of VTE. ② A VTE team was established to regularly discuss and summarize the problems during the prevention process, to resolve the nursing problems in practice by reviewing the literature, and to supervise the prevention process by the head nurse and a senior nurse.

### 3.1. Observation Criteria

1. General data: they included patients' gender, age, department of treatment, marital status, ethnic groups, education degree, occupation, hospitalization time, times of operation, and living habits.
2. Incidence of VTE: the study group received training to clarify the screening criteria of VTE. Patients were screened weekly after admission, which was also performed for patients with VTE symptoms. ① DVT assessment: D-D detection was performed for low-risk patients. If negative, they were excluded. If positive, venous ultrasound examination of the lower extremity will be performed to determine whether it was DVT. The same examination was firstly performed for middle-risk and high-risk patients. Treatment was given to positive ones, and the negative ones continued to be observed. ② PTE: low-risk and middle-risk patients were tested for the D-D level. Negative ones were excluded, and positive ones received CT pulmonary angiography (CTPA) examination (Philips, NMPA (I) certified no. 20083303600). If they were still positive, the diagnosis was confirmed, and treatment was started. CTPA examination was performed for high-risk patients. Negative ones were excluded, and positive ones received treatment. The total number of patients with VTE was recorded. VTE incidence = (DVT + PTE)/120 × 100.0%.
3. Scores of VTE awareness: the questionnaire of VTE awareness was formulated after reviewing the domestic and foreign literature and based on Guidelines of Venous Thromboembolism Prevention after Major Orthopedic Surgery in China [15], Chinese Prevention and Guidelines for Perioperative Thromboprevention [16], and Clinical Questionnaire of VTE prevention [17]. The questionnaire for patients was mainly about basic knowledge, with the scores of 0–100 points. Higher scores indicated higher awareness. The questionnaire for nursing staff included basic prevention, physical prevention, and drug prevention, with the scores of 23 points, each item for 1 point. The questionnaire for patients was used before and after nursing, and that for nursing staff was used at the beginning of the study and after nursing.
4. Nursing satisfaction: the self-made scale of our hospital was used to evaluate service quality, service attitude, and communication effectiveness, with total scores of 100 points for each item. Higher scores indicated higher satisfaction of patients.

### 3.2. Statistical Processing

In this study, the data were processed by SPSS 20.0 and graphed by GraphPad Prism 7 (GraphPad Software, San Diego, USA). Enumeration data were tested by *X*^2^ and expressed by frequency and percentage. Measurement data were tested by *t* and expressed by (‾*x* ± *s*). A test level of *α* = 0.05, and the differences were statistically significant at *P* < 0.05.

## 4. Results

### 4.1. Comparison of General Data

No significant difference was found in the general data of patients between both groups (*P* > 0.05) (see Table 1).

### 4.2. Comparison of the Incidence of VTE

Compared with the CG, the incidence of VTE of the OG was obviously lower (*P* < 0.05) (see Figure 2).

In the OG, numbers of cases with DVT, with PTE, and without VTE were 2 (3.3%), 0 (0.0%), and 58 (96.7%). In the CG, numbers of cases with DVT, with PTE, and without VTE were 6 (10.0%), 2 (3.3%), and 52 (86.7%).

### 4.3. Comparison of Scores of VTE Awareness of Patients and Nursing Staff

After nursing, compared with the CG, scores of VTE awareness in the OG were conspicuously higher (*P* < 0.001), and scores of VTE awareness of the nursing staff were conspicuously higher than those before nursing (*P* < 0.001) (see Figure 3).

### 4.4. Comparison of Nursing Satisfaction

Compared with the CG, nursing satisfaction of the OG was obviously higher (*P* < 0.001) (see Figure 4).

Compared with the CG, scores of service quality, service attitude, and communication effectiveness of the OG were obviously higher (92.65 ± 2.65 vs. 80.64 ± 3.68, 96.98 ± 1.52 vs. 84.98 ± 2.65, and 92.10 ± 1.68 vs. 80.68 ± 2.65, *P* < 0.001).

## 5. Discussion

Including DVT and PTE, VTE is one of the most common causes of death in medical inpatients, which can be prevented through suitable methods. According to foreign studies, without prevention care of the thrombus, the incidence of VTE in medical inpatients is 4.96%–50.0% [18], while that in Chinese studies is 9.7%–27.0%, and that in patients with congestive heart failure, stroke, and other diseases is up to 60.0% [19], indicating that VTE is an important factor affecting the life and health of patients. Previous studies have shown that the scientific and standardized VTE prevention measures can effectively reduce the incidence of VTE [20]. With the advance of medicine, medical staff pays much attention to VTE prevention, and more clinical nursing measures for VTE prevention are gradually emerging. However, the retrospective study conducted by Giancarlo et al. found that the effective prevention rate of VTE in hospitalized patients was not optimistic, and the proportion of patients who received appropriate VTE prevention measures was only 11.0%–19.0% [21]; therefore, it was crucial to improve the efficacy of VTE prevention measures.

In 2004 and 2008, the American College of Chest Physicians issued guidelines for VTE prevention, and the antithrombotic guidelines (2012) detailed the VTE prevention measures that should be taken in different situations, including VTE prevention in nonsurgical patients [22]. Chinese experts of VTE prevention have also drawn up various VTE prevention guidelines, but there is still no unified program in clinics. Hospitals try to build a suitable management system of thrombosis prevention according to VTE prevention experience, but it delivers little effect without the guidance of the SOP. On the basis of the original prevention plan, Shanghai Changhai Hospital revised the new version of VTE prevention guidelines [23]. Some scholars formulated the SOP for orthopedic DVT prevention based on Caprini risk assessment [24], which provided a reference for unifying the standard, but its clinical practicality still needed to be further explored. Through literature analysis and Delphi method, this study developed a scientific, standardized, reasonable, effective, and practical SOP for VTE prevention, with the main methods of learning from the key points of the domestic and foreign literature, combining with nursing experience, strengthening prevention management, training and education, and improving VTE assessment methods, so as to lower the incidence and mortality of VTE. At the end of the study, compared with the CG, the incidence of VTE in the OG was conspicuously lower (*P* < 0.05), indicating that the SOP of VTE prevention has good operability and can effectively reduce the incidence of VTE for patients.

Against the background of the laggard SOP of VTE in China and limited knowledge of some medical staff, the maximum effect of precautions cannot be achieved. In addition, without clear awareness of VTE, patients have poor prevention compliance. After systematic health education, awareness of VTE of patients and nursing staff was significantly deepened. Therefore, after nursing, compared with the CG, scores of VTE awareness in the OG were conspicuously higher (*P* < 0.001), and scores of VTE awareness of the nursing staff were conspicuously higher than those before nursing (*P* < 0.001), indicating that SOP could be cooperatively performed by both sides to improve the clinical practicability. Meanwhile, the incidence of VTE was lower and the nursing satisfaction was higher in the OG (*P* < 0.001), showing that SOP could reduce the nursing disputes. Bryce et al. found that nurse-patient communication was an important reason that impacted on the effect of nursing [25]. Therefore, in further study of the SOP of VTE prevention, it should focus on standard and detailed health education and communication for nursing staff, so as to full play the role of SOP of VTE prevention.

In conclusion, SOP can reduce the incidence of VTE of patients, improve their disease awareness, and enhance their nursing satisfaction, which should be popularized in practice.

## Figures and Tables

**Figure 1:** Flow diagram of the study.

**Figure 2:** Comparison of the incidence of VTE (*n* (%)). Note: the black area was DVT, the white area was PTE, and the grid area was no VTE. The OG was on the left, and the CG was on the right.

**Figure 3:** Comparison of scores of VTE awareness of patients and nursing staff (‾*x* ± *s*, points). (a) The scores of VTE awareness of patients. The abscissa was before and after nursing from left to right, respectively, and the ordinate was scores of VTE awareness (points). The black area was the OG, and the gray area was the CG. No significant difference was found in the scores of VTE awareness between both groups. After nursing, compared with the CG, the scores of VTE awareness in the OG were obviously higher (86.41 ± 2.68 vs. 72.11 ± 2.58, *P* < 0.001). (b) The scores of VTE awareness of nursing staff. The abscissa was basic prevention, physical prevention, and drug prevention from left to right, respectively, and the ordinate was scores of VTE awareness (points). The black area was at the beginning of the study, and the gray area was after nursing. After nursing, the scores of basic prevention, physical prevention, and drug prevention of nursing staff were obviously higher than those before (5.21 ± 0.42 vs. 4.04 ± 0.30, 10.98 ± 0.45 vs. 8.96 ± 0.45, and 4.56 ± 0.32 vs. 3.12 ± 0.62, *P* < 0.001).

**Figure 4:** Comparison of nursing satisfaction (‾*x* ± *s*, points). Note: the abscissa was service quality, service attitude, and communication effectiveness from left to right, and the ordinate was the scores of nursing satisfaction (points). The black area was the OG, and the gray area was the CG. # indicated *P* < 0.001.

**Table 1:** Comparison of general data.

Group	OG (*n* = 60)	CG (*n* = 60)	*X* ^2^/*t*	*P*
Gender			0.135	0.714
Male	32	34		
Female	28	26		
Age (years)				
Range	20–76	18–74		
Average age	48.98 ± 5.32	49.10 ± 5.36	0.123	0.902
Department				
Respiratory department	21	20	0.037	0.847
Department of cardiology	19	20	0.038	0.845
Department of neurology	9	10	0.063	0.803
Geriatric department	11	10	0.058	0.810
Marital status			0.344	0.558
Married	38	42	0.600	0.439
Unmarried, divorced, or widowed	22	18		
Ethnic groups			0.100	0.752
Han	55	54		
Ethnic minorities	5	6		
Education degree				
Primary school degree and below	21	20	0.037	0.847
Middle school	15	16	0.044	0.835
Junior college degree and above	24	24	0.000	1.000
Occupation				
Unemployment	12	15	0.430	0.512
Workers and peasants	32	30	0.134	0.715
Clerk	16	15	0.044	0.835
Hospitalization time (d)	52.68 ± 5.68	52.48 ± 5.21	0.201	0.841
Time of surgery	1.32 ± 0.21	1.30 ± 0.25	0.474	0.636
Living habits				
History of drinking	28	29	0.033	0.855
Smoking history	32	29	0.300	0.584

## Data Availability

The data used to support the findings of this study are available from the corresponding author upon reasonable request.
